RETRACTED

# The Combination Clinical Value of Plasma Brain Natriuretic Peptide and Serum HbAlc in the Diagnosis of Chronic Pulmonary Heart Disease

**DOI:** 10.1155/2022/6932179

**Published:** 2022-06-20

**Authors:** Enxia Jia

**Affiliations:** Department of Respiratory Medicine, Baoding Fourth Central Hospital, Hebei Province, China

## Abstract

**Objective:**

To analyze the combination clinical value of plasma brain natriuretic peptide and serum glycated hemoglobin (HbAlc) in chronic pulmonary heart disease.

**Methods:**

A total of 200 patients with chronic pulmonary heart disease admitted to our hospital from January 2021 to January 2022 were selected as the observation group, and 200 healthy subjects were selected as the control group during the same period. All subjects were examined by an ECG vector map and plasma BNP, and HbAlc levels were detected to analyze the value and clinical significance of each index in single diagnosis and combined diagnosis.

**Results:**

Plasma BNP and HbAlc levels in the observation group were significantly higher than those in the control group (*P* < 0.05). There were 154 BNP positive, 146 HbAlc positive, 164 parallel combined diagnosis positive, and 132 serial combined diagnosis positive. Sensitivity of series combination diagnosis was significantly higher than other indexes (*P* < 0.05); especially, parallel combination diagnosis was significantly higher than other indexes (*P* < 0.05). Besides, area under the ROC curve of parallel combination diagnosis and series combination diagnosis was significantly higher than that of each index alone diagnosis (*P* < 0.05).

**Conclusion:**

In the diagnosis of chronic pulmonary heart disease, the combination of plasma BNP and HbAlc can effectively improve the diagnostic specificity and sensitivity, as well as improve the area under the ROC curve.

## 1. Introduction

Chronic pulmonary heart disease, also known as cor pulmonale in clinic, is a common disease of the respiratory system in middle-aged and elderly people in China [1]. Clinical research has shown that in patients with various kinds of organic heart disease, about 20%~40% are pulmonary heart disease, and with the progress of patients' disease, it is likely to induce many complications, causing serious adverse effects on the quality of life and life safety of patients [2]. Studies have found that the pathogenesis of patients with cor pulmonale is mainly due to pulmonary vascular disease or vascular disease of the branch air duct and lung tissue, which causes the increase of pulmonary arterial blood pressure and then leads to heart disease [3–5]. Clinically, patients are often divided into chronic pulmonary heart disease and acute pulmonary heart disease according to their disease status. Chronic pulmonary heart disease is the most commonly occurred [6]. Under normal circumstances, the onset of pulmonary heart disease is slow; early detection and timely treatment of pulmonary heart disease can reduce the failure of cardiopulmonary function and other organ damage [7–9]. At present, ECG, X-ray, and ultrasonic examination are often used in the diagnosis of patients with pulmonary heart disease. The electrocardiogram showed right ventricular hypertrophy, peaked P wave, and arrhythmias. And the chest X-ray showed the prominent pulmonary vessels, right atrial dilation, and right ventricular hypertrophy [10]. However, pulmonary heart disease is easily confused with bronchitis, so imaging combined with serology can be used in clinical diagnosis [11–13].

RETRACTED

Chronic pulmonary heart disease is referred to as pulmonary heart disease [14]. Pulmonary heart disease refers to chronic pulmonary chest disease or chronic pulmonary vascular disease, which gradually causes pulmonary hypertension and then causes right ventricular hypertrophy and finally a heart disease of heart failure [15]. It is a common and frequently occurring disease. As a common clinical pulmonary disease, heart pulmonale disease is increasing, due to the increasing life pressure and environmental deterioration in recent years [16]. If pulmonary heart disease is not treated with effective measures in time, the disease will worsen year by year, which will bring a great threat to the patient's physical and mental health and life safety. This is particularly critical in the early stage of accurate diagnosis and effective treatment of chronic pulmonary heart disease [17]. Now, the diagnosis of chronic cor pulmonale relies on more clinical electrocardiogram (ECG), colour to exceed, X-ray inspection, and physicians according to patients' symptoms, history of disease and symptoms, and diagnosis, but as a result of the clinical manifestations of chronic cor pulmonale with diverse and special sex, especially for patients with early stage and elderly patients, often, there are complications and it increased the difficulty of the clinical diagnosis [18]. Pulmonary hypertension will ultimately lead to abnormal lung function; pulmonary disorders occur, as the main pathogenesis of cor pulmonale. Studies about the disease in recent years have shown that there is a close relationship between pulmonary artery high-pressure forming process and a variety of vascular active substances. The main function is to adjust pulmonary circulation function, which is given priority with plasma BNP [19].

The purpose of this study was to analyze the diagnostic value and clinical significance of plasma brain natriuretic peptide (BNP) combined with glycated hemoglobin (HbAlc) in patients with chronic pulmonary heart disease treated in our hospital.

RETRACTED

## 2. Materials and Methods

### 2.1. General Information

A total of 200 patients with chronic pulmonary heart disease admitted to our hospital from January 2021 to January 2022 were selected as the observation group, and 200 healthy physical examination subjects during the same period were selected as the comparison group. There were 168 males and 132 females in the observation group, with an age of 65.83 ± 9.89 years and a course of disease of 16.68 ± 5.92 years. There were 166 males and 134 females in the control group, aged 66.19 ± 10.05 years. The significance of the selection of the control group was considered as a control. There are no missing patients in the enrollment process. There was no statistical difference between the two groups (*P* > 0.05). The study was approved by our ethics committee.

### 2.2. Inclusion Criteria

The inclusion criteria are as follows: (1) the observation group had a family history of lung disease; (2) diagnosed by imaging examination, including X-ray and computerized tomography (CT); (3) age older than or equal to 18; and (4) informed about the study and signed informed consent.

### 2.3. Exclusion Criteria

The exclusion criteria are as follows: (1) congenital heart disease and chronic constrictive pericarditis; (2) primary cardiomyopathy and rheumatic heart disease; (3) rheumatic heart valve disease; and (4) voluntarily apply for withdrawal from the study.

### 2.4. Detection Method

All subjects in this study were examined by ECG vector maps and by SE-1515 ECG workstation, and an electrode was placed according to the Frank lead system. Fasting venous blood was collected, and serum BNP and HbAlc levels were measured by an enzyme-linked immunosorbent test. All the kits used were purchased from Lianke Biotechnology, and all operations were performed in strict accordance with the kit instructions.

### 2.5. Diagnostic Criteria

HbA1c ≥ 6.1% and BNP ≥ 100 pg/mL were considered as positive. In parallel combination and series combination during joint diagnosis, if any indicator is positive, the parallel diagnosis is considered positive, if all indicators are positive, and the serial combined diagnosis was determined to be positive.

### 2.6. Statistical Analysis

SPSS 23.0 was used for statistical analysis, measurement data were expressed as *X* ± *S*, *t*, counting data were expressed as percentage table, *t*, pathological diagnosis was used as the gold standard, ROC curve was drawn to analyze the diagnostic efficacy of each indicator diagnosis, and *P* < 0.05 was considered statistically significant.

RETRACTED

## 3. Result

### 3.1. Test Results of Each Indicator

There were statistically significant differences in ECG vector mapping between the two groups, and the levels of BNP and HbAlc in the observation group were significantly higher than those in the contrast group (*P* = 0.001) (Table 1).

### 3.2. Diagnostic and Evaluation Results of Each Index

83 were positive for ECG charts, 85 for BNP, 81 for HbAlc, 95 for parallel combinations, and 79 in series (Table 2).

### 3.3. Results of the Diagnostic Efficacy Assessment of Each Index

The results of this group showed that the combined diagnosis sensitivity of series was significantly higher than other indicators (*P* < 0.05), and the parallel combination diagnosis specificity was significantly higher than other indicators (*P* < 0.05) (Table 3), and the area under the ROC curve of parallel combination and series combined diagnosis was significantly higher than that of each index (*P* < 0.05) (Figure 1).

### 3.4. Treatment of Chronic Pulmonary Heart Disease in Two Groups

Two groups of patients with severe acute pulmonary heart disease were treated with a high-flow humidified oxygen therapy apparatus (Airvo, Fisher & Paykel Healthcare, LTD), using a double-cavity nasal catheter oxygen inhalation; the initial temperature was 37°C; the oxygen concentration was 35%; the flow rate was adjusted to 30-50 L/min; and the treatment time > 6 h. Humidification treatment parameters were adjusted according to the blood gas index of vital sign instrument, and blood oxygen saturation ≥ 90%. The treatment cycle was 3 days, and catheterization was carried out in time if the patient's condition deteriorated (Figure 2).

## 4. Discussion

In recent years, with the change of people's lifestyle and environmental deterioration, the incidence of clinical pulmonary heart disease is increasing year by year [20]. In a variety of visceral heart disease, about 20%~40% are pulmonary heart disease [21–24]. Pulmonary heart disease is mostly induced by chronic obstructive pulmonary disease, and it is a slow occurrence and development process [25]. If the condition is not controlled in time, it may lead to right heart failure, leading to the death of end-stage patients. ECG vector graph is a widely used detection technique in clinical practice in recent years, which is mainly used to detect the electrical activity of the cardiac cycle in subject changes. It has the advantages of simple operation and wide application. However, with the significant development of human diseases and the improvement of medical technology, the effect of traditional electrocardiogram still needs to improve [26–29]. ECG vector chart can effectively record the size and direction of electrical signals generated by the heart, effectively eliminate all kinds of heart diseases except arrhythmia, and truly and effectively describe the stereoscopic image of heart activity. This method is used to diagnose heart disease, improve the effectiveness of clinical diagnosis, and make up for the insufficient diagnosis of ventricular hypertrophy by traditional electrocardiogram. Brain natriuretic peptide is a peptide hormone secreted mainly by the left ventricle [30]. It has the effects of natriuretic, diuretic, vasodilator, antihypertensive, and antagonistic against renin J angiotensin J aldosterone system activity. The increase of pressure and tension of left ventricular wall can promote its secretion, which can reflect the change of left ventricular function sensitively and specifically. At present, it is mainly used in the diagnosis and prognosis evaluation of left ventricular dysfunction [31]. The results showed that the level of brain natriuretic peptide in acute exacerbation and remission stage of cor pulmonale was higher than that in the control group, suggesting that brain natriuretic peptide was also involved in the pathophysiological process of right ventricular changes in cor pulmonale [32]. The level of brain natriuretic peptide in acute exacerbation stage was the highest but decreased in remission stage, but it was still higher than that in the control group, suggesting that brain natriuretic peptide can be used as one of the indicators to judge the severity of pulmonary heart disease.

RETRACTED

After binding with its receptor, BNP can effectively activate intracellular guanosine cyclase, synthesize cGMP to play biological effects, achieve antidiuretic, inhibit sympathetic nervous activity, reduce pulmonary circulation, inhibit the antirenin angiotensin system, reduce peripheral circulation vascular tension ability, and effectively dilate blood vessels [33]. BNP has a short half-life and is catabolized by neuronal peptidase. BNP can also be metabolized by the intracellular lysosomal system by binding to receptors and transferring into cells. In physiological state, the human body will also synthesize and secrete BNP, but its level is far lower than many pathological conditions. Studies have pointed out that when the heart load is too heavy or the heart chamber is pulled, increasing the internal pressure of the heart, releasing the ventricular BNP, reducing the heart load, improving the heart function, reducing the systemic circulation resistance, and maintaining the normal function and structure of the heart have a very important role [34, 35]. HbAlc is a ketone ammoniated compound formed by n-acetylglucosamine and *β*-terminal amino acids after the synthesis of hemoglobin in the human body. Some studies have pointed out that blood glucose level is a decisive factor in determining the amount of HbAlc. In general, the formation time of hBA1c is longer and the formation stability of HBA1C is higher. Studies have pointed out that patients with cor pulmonale suffer from impaired lung function, resulting in lower body parameters than healthy people. Due to the decrease of blood oxygen concentration and obstruction of the respiratory tract, HbAlc level in patients is increased, and the increase of water level may lead to further decrease of lung function.

RETRACTED

In conclusion, the combination of plasma brain natriuretic peptide and HbAlc in the diagnosis of chronic pulmonary heart disease can effectively improve the diagnostic specificity and sensitivity and improve the area under the ROC curve. However, the clinical sample size of this study is small, which requires further study to expand the clinical sample size.

## Figures and Tables

**Figure 1:** POC curve evaluation and analysis.

**Figure 2:** (a–d) Treatment of chronic pulmonary heart disease patients. (a) The X-ray of the chronic pulmonary heart disease. (b) The computerized tomography (CT) of pulmonary heart disease. (c, d) Patients were treated with a high-flow humidified oxygen therapy instrument.

**Table 1:** Test results of each index.

Groups	Cases (*N*)	Monocardiogram (*N*)		BNP (pg/mL)	HbA1c (mg/dL)
		Normal	Abnormal		
Experimental group	200	67	143	108.85 ± 4.85	8.75 ± 2.15
Control group	200	143	57	38.18 ± 6.25	7.85 ± 1.35
*t*	—	58.315		58.845	8.385
*P*	—	0.001		0.001	0.001

**Table 2:** Diagnosis and evaluation results of each index (*n*).

Groups		Pathologic diagnosis		Total
		(+)	(-)	
Monocardiogram	(+)	83	13	96
	(-)	19	85	104

BNP	(+)	85	19	104
	(-)	13	83	96

HbA1c	(+)	81	15	96
	(-)	19	85	104

Parallel combined inspection	(+)	95	19	104
	(-)	5	81	86

Serial combined inspection	(+)	79	3	82
	(-)	123	195	318

Total		200	200	

**Table 3:** Results of the diagnostic efficacy assessment of each index.

Groups	Sensitivity (%)	Specificity (%)	ROC area under the curve
Monocardiogram	85.45	83.68	0.751
BNP	82.68	85.45	0.715
HbA1c	83.35	81.75	0.875
Parallel combined inspection	82.55	93.01	0.889
Serial combined inspection	95.15	82.38	0.932

## Data Availability

The data used to support this study are available from the corresponding author upon request.
